# The Role of Allograft Inflammatory Factor-1 in the Effects of Experimental Diabetes on B Cell Functions in the Heart

**DOI:** 10.3389/fcvm.2018.00126

**Published:** 2018-09-11

**Authors:** Amrita Sarkar, Sanket K. Shukla, Aseel Alqatawni, Anil Kumar, Sankar Addya, Alexander Y. Tsygankov, Khadija Rafiq

**Affiliations:** ^1^Center for Translational Medicine, Thomas Jefferson University, Philadelphia, PA, United States; ^2^Department of Microbiology and Immunology, Thomas Jefferson University, Philadelphia, PA, United States; ^3^Kimmel Cancer Centre, Thomas Jefferson University, Philadelphia, PA, United States; ^4^Microbiology and Immunology, Lewis Katz School of Medicine, Temple University, Philadelphia, PA, United States

**Keywords:** diabetic cardiomyopathy, inflammatory responses, B cells, allograft inflammatory factor-1, Streptozotocin (STZ), type 1 diabetes (T1D)

## Abstract

Diabetes mellitus (DM) often causes chronic inflammation, hypertrophy, apoptosis and fibrosis in the heart and subsequently leads to myocardial remodeling, deteriorated cardiac function and heart failure. However, the etiology of the cardiac disease is unknown. Therefore, we assessed the gene expression in the left ventricle of diabetic and non-diabetic mice using Affymetrix microarray analysis. Allograft inflammatory factor-1 (AIF-1), one of the top downregulated B cell inflammatory genes, is associated with B cell functions in inflammatory responses. Real-time reverse transcriptase-polymerase chain reaction confirmed the Affymetrix data. The expression of CD19 and AIF-1 were downregulated in diabetic hearts as compared to control hearts. Using *in vitro* migration assay, we showed for the first time that AIF-1 is responsible for B cell migration as B cells migrated to GFP-AIF-1-transfected H9C2 cells compared to empty vector-transfected cells. Interestingly, overexpression of AIF-1 in diabetic mice prevented streptozotocin-induced cardiac dysfunction, inflammation and promoted B cell homing into the heart. Our results suggest that AIF-1 downregulation inhibited B cell homing into diabetic hearts, thus promoting inflammation that leads to the development of diabetic cardiomyopathy, and that overexpression of AIF-1 could be a novel treatment for this condition.

## Introduction

Diabetes is a metabolic disorder whose primary manifestation is the elevated level of circulating blood glucose. It can be caused by either insulin deficiency (type 1 diabetes) or insulin resistance (type 2 diabetes). Clinical, epidemiological, and experimental studies all point to the existence in diabetes a cardiac dysfunction independent of hypertension and underlying coronary artery disease (1, 2). This deterioration in heart function, known as diabetic cardiomyopathy (DCM), is frequently associated with alterations in myocardial calcium handling, premature myocyte death and impaired ventricular function that ultimately leads to adverse cardiac remodeling and congestive heart failure (3–9). Cardiovascular disease (CVD) is the most prevalent cause of morbidity and mortality in diabetic patients (10, 11). In the absence of knowledge about the disease-specific mechanisms responsible for cardiomyocyte death, the design of appropriate and effective interventions and strategies for the prevention of CVD in diabetes has been challenging.

Studies that have been performed in order to understand the basis of altered myocardial structure and function in DCM are not controversial or questionably designed, but they simply have not evolved to provide sufficient mechanistic insight related to involvement of inflammatory responses as a pathophysiological trigger. Recently, increasing evidence suggested that the B cell-mediated immunity plays an important role in cardiac dysfunction in diabetic mice (12). However, the role of B cells in the onset of DCM and in its preclinical manifestation—diastolic dysfunction—has not been unraveled so far. During inflammation, the B cell antigen receptors bind to the corresponding antigens and internalize them (13). Under normal conditions, B cells differentiate to produce antibodies, which are involved in the function of innate immunity as well, and to yield memory cells to effectively respond to future challenges by the same antigens (13). B cells play a crucial role in maintaining the bridge between innate and adaptive immunity (14–16). During inflammation, B cells sense exogenous inflammatory triggers that activate toll-like receptors thus promoting the crosstalk between innate and adaptive immunity (17, 18). Previously, it has been shown that B cells play a key role in the development of various autoimmune conditions (19). However, the exact mechanism by which B cells regulate heart functions during the development of DCM remains unknown. Therefore, the need to investigate new pathogenic mechanisms involved in the course and progression of this devastating disease is urgent; these mechanisms must be explored in order to develop alternative therapeutic strategies.

It is well recognized that patients with diabetes are more prone to infection and inflammation (20). Shoelson et al. (21) reported the association of inflammation with the carbohydrate metabolism and insulin level. B cells influence and regulate the immune response by several mechanisms and represent a complex, but important link between the innate and adaptive immune systems (22–25). B cells are not only central to the production and amplification of humoral immune responses, but also play an important role as antigen-presenting cells, thereby contributing to the maintenance of immune tolerance, as well as a regulatory role in inflammation (19, 26). To advance the specific goal for the resolution of inflammation in cardiac healing, it is necessary to understand leukocyte diversity and the milieu around leukocytes in cardiac pathology, particularly in the context of obesity and diabetes. Thus, targeting B cell phenotype may be a novel developing topic in cardiac recovery. Our finding suggested that one of the molecules associated with the B cell function during inflammatory response is allograft inflammatory factor-1 (AIF-1). AIF-1 is a cytokine with calcium (Ca^++^)-binding EF-hand domains, which is constitutively expressed in lymphatic tissue (27) and has been reported to enhance the activation of lymphocytes (28). AIF-1 appears to play a fundamental role in several cell types involved in chronic immunological inflammatory processes, especially macrophages. In particular, its expression is up-regulated in monocytes/macrophages under various pathological conditions (29, 30) and its synthesis can be induced by interferon-γ (29). Moreover, AIF-1 is expressed by microglial cells following cerebral infarction (31) and by the glandular and stromal cells of endometrial tissues in endometriosis (32). However, no study has shown the effect of AIF-1 on B cell homing into the hearts during the development of DCM.

In this study, we investigated the possible association between the B cell homing to heart tissues and AIF-1 expression during the development of DCM. We found that diabetes-induced heart dysfunction was associated with a decrease in the numbers of B cells as well as in AIF-1 expression in heart tissues. Interestingly, our *in vitro* and *in vivo* data showed that AIF-1 plays a role in B cell migration to cardiomyocytes. Hence, these findings reveal a hitherto unidentified role for AIF-1 expression in B cell immunity and cardiac function that may provide important insight into preventing or delaying cardiac diseases during the progression of diabetes.

## Materials and methods

### Experimental animals

Wild-type (WT) C57BL/6 male mice, 8 weeks of age, were purchased from the Jackson Laboratory (Bar Harbor, Maine). Mice were housed at Thomas Jefferson University at 22°C with a 12 h light/dark cycle with free access to standard rodent chow and tap water. All animal protocols have been approved by the Institutional Animal Care Committee of Thomas Jefferson University, and experiments conformed to the Guide for the Care and Use of Laboratory Animals published by the U.S. National Institutes of Health and approved by the American Physiological Society. All the methods were carried out in accordance with the relevant guidelines and regulations.

### Induction of diabetes in mice

Type 1 diabetes-like condition was induced in 8-week-old (8W) old mice by intraperitoneal injection of streptozotocin (STZ) [Sigma-Aldrich, St. Louis, MO, dissolved in 0.1 M sodium citrate (pH 4.5)] at a dose of 50 mg/kg body weight for 5 consecutive days, while age-matched control mice received sodium citrate buffer injection in the same manner. This strategy minimizes nonspecific toxic effects of high-dose STZ and also provides a robust and consistent hyperglycaemic response in mice model (33–38). We labeled two groups of mice: STZ-treated WT mice and WT control mice. After 5 days of last injection of STZ, mice with blood glucose levels ≥250 mg/dl (13.88 mM) were defined as diabetic as described previously (39). HbA_1c_ levels were measured at each end point of the study using standard kit (Crystal Chem USA). At 4 and 8 W after STZ injection, mice were sacrificed for experimental measurements using intraperitoneal injection of anesthesia (xylazine: ketamine: water = 1:2:3) (40–43). To evaluate whether STZ has any toxic effect on the mouse heart, we used OVE26 mice, a genetic mouse model of type 1 diabetes, overexpressing a calmodulin mini-gene under the control of the rat insulin II promoter that develops specific islet ß-cell destruction, thus leading to severe and consistent insulin-deficient diabetes with an early onset of hyperglycemia.

### Echocardiographic measurement

Cardiac function and ventricular dimensions were assessed by echocardiographic measurement before STZ injection as well as at 4 and 8 W after STZ injection before sacrifice. Briefly, following light sedation with 1% isoflurane, mice were placed on a platform in left lateral decubitus position for imaging. The isoflurane gas volume was regulated according to the rate in order to ensure an adequate depth of anesthesia. All the hairs were removed from chest area using chemical hair remover, and aquasonic clear ultrasound gel (Parker Laboratories, Fairfield, NJ) without bubbles was applied to the thorax surface to optimize the visibility of the cardiac chambers. Echocardiography was done using Visualsonic Ultrasound System (Vevo770, Toronto, Canada) containing a 40 Mhz variable frequency probe. Standard imaging planes, M-mode, color-mode, Doppler, PW Doppler mode views were recorded when the mouse possessed a target heart rate between 450 and 550 beats per minute (44). Functional calculations were acquired according to the guidelines of the American Society of Echocardiography. Heart rate, percent ejection fraction (%EF), percent fractional shortening (%FS), LV diastolic posterior wall thickness, LV systolic posterior wall thickness, intraventricular diastolic septum thickness, intraventricular systolic septum thickness, LV diastolic internal diameter, LV systolic internal diameter, E wave velocity, A wave velocity, mitral peak velocity of early filling (E) to mitral peak velocity of late filling (A) E/A ratio, Isovolumic Relaxation Time IVRT, LV mass, LV mass (corrected), LV diastolic volume, LV systolic volume, Left ventricular (LV) mass, and heart weight/tibia length were calculated (45). muMT 8W (B cell knock out) mice with or without STZ injection were used to show as a negative control here to prove that STZ leads to the development to DCM in the absence of B cells.

### Microarray

Total LV heart RNA was isolated from STZ-treated WT and age-matched control mice at 4 and 8 W. RNA isolation was done using RNeasy mini kit (Qiagen, Mansfield, MA) according to the manufacturer's instructions. Fragmented biotin-labeled cDNA (from 100 ng of RNA) was synthesized using the GeneChip WT PLUS reagent kit (Affymetrix, Santa Clara, CA). The protocols for microarray experiments were previously described (46). In brief, we hybridized each Affymetrix GeneChip Mouse 2.0 ST array with fragmented and biotin-labeled target (4.5 μg) in 200 μL of hybridization cocktail. Target denaturation was performed at 99°C for 5 min and then at 45°C for 5 min followed by hybridization for 16 h at 45°C. Next the arrays were washed and stained using GeneChip Fluidic Station 450 using the Affymetrix GeneChip hybridization wash and stain kit. Chips were scanned on the Affymetrix GeneChip Scanner 3000 7G using Command Console Software. Quality control of the experiment was done by Expression Console Software V 1.4.1. Data were analyzed using GeneSpring software 14.8 (Agilent Technologies, Inc., Santa Clara, CA). The probe set signals were calculated with the Iterative Plier 16 summarization algorithm; baseline to median of all samples was used as baseline option. The criteria for differentially expressed genes were set at ≥ 1.5-fold change. Statistical analysis was performed to compare two groups using the unpaired *t*-test with *p*-value < 0.05 considered statistically significant. Heat maps were generated from differentially expressed gene list.

### Ingenuity pathway analysis (IPA)

The list of differentially expressed genes was loaded into the Ingenuity Pathway Analysis (IPA) 8.0 software (http://www.ingenuity.com) to perform biological network and functional analysis.

### Immunohistochemistry

Tissues were fixed in 10% formalin, embedded in paraffin, and sectioned at 6 μm thickness. Paraffin heart sections were deparaffinised in xylene and rehydrated. Antigen retrieval was achieved by boiling the slides in citrate solution for 20 min, and slides were then washed with phosphate-buffered saline (PBS). After quenching endogenous tissue peroxidase activity with 3% H_2_O_2_ for 15 min, slides were washed in PBS and blocked in PBS containing 2.5% serum at room temperature for 30 min. Primary antibodies to detect CD19 (Cell signaling, 3,574 s) and CD21 (Abcam, ab75985) were applied in PBS containing 2.5% serum for overnight incubation at 4°C. The next day, samples were washed in PBS and then sequentially incubated with Vectastain Elite ABC Kit (Avidin/Biotin/Horseradish Peroxidase-System, Vector Laboratories). The peroxidase reaction was visualized using 3,3′-diaminobenzidine tetrahydrochloride (DAB), and slides were counterstained with haematoxylin. All the images were captured at 40X magnification using bright field microscope. Cells were counted using Image J by adjusting to a lower and upper (Pixel) threshold (Image, Adjust, Threshold, Set or Auto). Then using the analyze particle tool (Analyze, Analyze Particles), the number of spots which implies the specific staining positive cells was counted automatically.

### Immunoblot analysis

Extraction of proteins from heart tissue samples was performed as follows. The heart tissues were homogenized, and cell lysates were obtained in FAK lysis buffer (50 mM Tris-HCl, pH 7.5, 100 μM sodium pyrophosphate, 1 mM sodium fluoride, 150 mM NaCl, 0.1% SDS, 1% triton X-100, 0.5 mM EDTA) containing inhibitors. The lysates were cleared by centrifugation, and the supernatants were subjected to immunoblotting analysis according to the manufacturers' instructions. Each panel in each figure represents results from a single gel exposed for a uniform duration, with bands detected by LI-COR Odyssey imaging system (PCSH898; LI-COR, Inc., Nebraska USA).

#### Cell isolation and flow cytometry

Lymphocytes were isolated from the heart by rinsing blood cells off with PBS. Heart tissue, minced into small pieces, was then digested in HBSS containing Ca^2+^, Mg^2+^, 25 mM HEPES buffer, 0.2 mg/ml DNAse I (Roche) and 12.5 μg/ml Liberase TM (Roche) under stirring at 37°C for two subsequent 30 min incubations. Released cells were filtered from the buffer after each incubation step through a 100-μm cell strainer, immediately washed with media containing serum and kept on ice (47, 48).

Two million cells per sample were stained for flow cytometry. To reduce nonspecific staining, cells were resuspended in 10 μL of Fc block (rat IgG and anti-FcγRII/III clone 2.4G2) and Aqua Blue Live/Dead Fixable Dead Cell Stain (Thermo Fisher Scientific) in staining buffer (PBS containing 0.2% BSA) for 2 to 5 min. After blocking, the cells were labeled with Alexa Fluor 700A-conjugated CD45 (clone RA3-6B2 103239, Biolegend) and PE-Cy7-conjugated CD19 (clone 1D3; ebio, 25-0193-82). Samples were acquired on a BD LSRII flow cytometer (BD Biosciences) and analyzed using FlowJo software (Tree Star, Ashland, OR). Dead cells were excluded from the analysis.

### Quantitative real-time PCR

cDNA was generated from RNA, and real-time PCR assays were performed using QuantiTect SYBR Green PCR kit (Qiagen, Crawley, UK) with specific primers to analyse the expression of TNF-α, IL-6, IL-1β, IL-4, IL-21, and AIF-1. PCR primers were bought from Life Technologies (CA, USA). The cycle threshold (*C*_*t*_) values of the target genes were first normalized to the *C*_*t*_ values of endogenous control GAPDH, an endogenous control. The results were plotted as normalized values.

### Immunofluorescence

CD19/α-actinin and AIF-1/α-actinin staining was done with the paraffin-embedded tissue sections to assess the co-localization. The tissue sections were fixed with 4% paraformaldehyde, washed with PBS and blocked with 2% BSA. The cells were then incubated with the first primary antibody at 4°C overnight. After repeated wash with PBS, the cells were incubated with Alexa Fluor 594 secondary antibodies. The fixed tissues were again washed with PBS and incubated with the second primary antibody that was biotinylated at 4°C overnight. Next day, an Alexa Fluor 488 streptavidin probe was added to the section and incubated for 1h and then washed away with PBS. The fluorescent stain 4′,6-diamidino-2-phenylindole (DAPI; 1:3,000 dilution) was added for 10 min, and the samples were mounted with DAKO mounting media (Agilent Technologies, S302380-2). The slides were visualized using an epifluorescence microscope (Leica Microsystems, Bannockburn IL) and images were captured at 40X magnification.

### Culture of H9C2 cardiomyocyte and A20 B cell lines

H9C2 cell line was purchased from ATCC, VA, USA and plated in 25 mm^2^ area of flask using DMEM media containing 10% heat inactivated (HI) fetal bovine serum (FBS) and antibiotic/antimycotic solution. A20 cell line was also purchased from ATCC and plated in 25 mm^2^ area of flask using RPMI media containing 10% HI-FBS, antibiotic/antimycotic solution. Every 2 days, cells were passaged and incubated at 37°C under 95% humidity with 5% CO_2_.

### Preparation of vectors

#### AIF-1-GFP plasmid preparation

The full-length mouse AIF-1 cDNA was PCR-amplified and inserted into the *KpnI-Not*I sites of the pCMV6-AC-GFP vector (Origene, MD, USA). After transformation to *E. coli* DH5α strain, clones were selected on solid LB media containing 50mg/L ampicillin. Multiple colonies were screened by colony PCR. After selecting the positive recombinant pCMV-AC-GFP-AIF-1, the plasmid DNA was extracted from the overnight culture and confirmed by the restriction digestion with *Kpn*I and *Not*I enzymes.

#### AdAIF-1 preparation

The full-length mouse AIF-1 cDNA was PCR-amplified and inserted into the *Kpn*I-*Xho*I sites of the pShuttle-CMV vector (Agilent Technologies). Recombinant AIF-1-expressing adenovirus AdAIF-1 was produced by homologous recombination of pShuttle-CMV-AIF-1 with the pAdEasy-1 adenoviral vector (Agilent Technologies) in *E.coli* strain BJ5183 according to the manufacturer's instructions. The AdAIF-1 was amplified in 293T cell line (ATCC). The titer of virus stock was determined by a plaque assay described by Tollefson et al. (49).

### Migration study

The H9C2 cells were plated in the lower chamber of a 8μm pore size transwell permeable support plate in DMEM media plus antibiotics/antimycotics with 10% FBS. On the next day, those cells were transfected either with GFP-tagged AIF-1 plasmid (5 μg/well) or a GFP-empty vector (transfection reagent was bought from Clonetech, Takara, CA, USA). In the meantime, A20 B cells were transfected with a RFP-empty vector in RPMI media containing 10% HI-FBS and antibiotic/antimycotic solution for 48h. When RFP transfection was confirmed, A20 B cells were replated in the upper chamber of the transwell plate. H9C2 and A20 B cells were incubated in fresh serum free DMEM media supplemented with antibiotic/antimycotic solution. Migration was observed at several time points: 1, 2, 4, and 8 h.

### AdAIF-1 injection to diabetic mice

To overexpress AIF-1 gene in mice we used the adenovirus expression system. Four groups of mice were studied: WT control, WT STZ 8W, mGFP-AdAIF-1-injected WT control and mGFP-AdAIF-1-injected WT STZ 8W. We mainly focused on STZ 8W mice, as the data showed a significant increase in the cardiac dysfunction and inflammatory responses followed by downregulation of B cells at 8W as compared to what was observed in WT STZ 4 W. Two weeks after diabetes induction, the mGFP-AdAIF-1 (mouse GFP tagged-AIF-1 adenovirus) (genecopoeia, Rockville, MD, USA) was injected intravenously at every alternative 2 weeks (1.5 × 10^8^ IFU/day; 200 ul). At 8 W after STZ injection, echocardiography was performed, mice were sacrificed, and tissues were collected for histology, PCR and immunoblot analysis. Untreated control and STZ mice also received empty factor too as control. We didn't show the result because they are the same as normal control.

#### Statistical analysis

Data analysis was performed using Origin pro version 8.5.1 software followed by GraphPad Prism 6 software (La Jolla, California, USA). All analyses represent at least three independent experiments and each time sample size *n* = 6 (for echo *n* = 12) and are expressed as mean ± standard error of the mean (SEM). Data from using chamber experiments were analyzed using one-way ANOVA without repeated measures when comparing more than two groups; Dunnett post-tests were used when comparing all treatments to control value only, and Tukey's post-tests were used when comparing treatments to control and other treatment values. One-sample *t*-tests were used when comparing a treatment value to a hypothetical control value (100%), student *t*-tests were used to compare two groups. For microarray data, Data analyses were performed by using GeneSpring software version 14.5 (Agilent Technologies, Inc., Santa Clara, CA). A paired *t*-test compared the “before” and “after” treatment samples. A statistical threshold of *p* < 0.05 with fold-change (FC) ≥ 1.5 was considered as significant for identification of differentially expressed genes. The probe set signals were calculated with the Iterative Plier 16 summarization algorithm; baseline to median of all samples was used as baseline option. For the western blotting time-course experiment, ratios of phosphorylated protein to total protein densitometry values were calculated and analyzed using one-way ANOVA and Dunnett post-test. For western blotting inhibitor studies, ratios of phosphorylated protein to total protein densitometry values were calculated then normalized to total fluorescence of blot to account for variation between experiments. A *p*-value of less than 0.05 (*p* < 0.05) was considered to be a significant difference. In table legend, ^*^ means Ctrl data were similar at 4 and 8 W, ^#^ means STZ 4W vs STZ 8W. Therefore, we showed only 1 control.

## Results

### Deterioration of cardiac structure and function in diabetic mice

We first monitored changes in body weight and blood glucose level in control and STZ-injected mice throughout the experimental period. In our study, STZ-treated WT mice showed severe hyperglycaemia (>250 mg/dL or 13.88 mM) already 1 week after the STZ injection (data not shown) and sustained it at 4 and 8 W, while the glucose level in normal mice consistently remained below 250 mg/dL (13.88 mM) (Table 1). HbA_1c_ also confirmed the induction of diabetes in mice model in the being of the experiment at each time point (Table 1). Further, STZ-treated mice exhibited the lower body weight as compared to the control group as previously reported (Table 1) (33, 39). To determine whether STZ induced cardiac dysfunction in WT mice, we examined cardiac function using echocardiography. Ultrasound echocardiography assessment demonstrated that the STZ treatment resulted in a progressive increase in left ventricular (LV) mass, left ventricular end diastolic diameter and heart weight/tibia length at 4 W, and these parameters further increased at 8 W. Ejection fraction (EF), fraction shortening (FS), IVRT, E/A ratio and other parameters from echocardiography measurements were significantly altered in the diabetic groups at 4 and 8 W as compared to the control group (Table 1). OVE26 mice were used as a positive control to STZ model, show an increase in blood glucose level and a decrease in body weight and cardiac contractile function (Table 1).

**Table 1:** Physiological parameters and echocardiography assessment of heart function after diabetes induction.

**Parameters**	**WT**			**OVE26**
	^*^Ctrl	**STZ 4W**	**STZ 8W**	
BG (mg/dl) or BG (mM)	128.0 ± 16.23 or 7.10 ± 1.89	482.0 ± 13.24^*^ or 26.751 ± 1.37	584.0 ± 10.17^*^^#^ or 32.41 ± 1.24	601.0 ± 21.04^*^ or 33.36 ± 2.18
BW (g)	26.0 ± 3.15	23.0 ± 2.28^*^	18.0 ± 2.25^*^^#^	17.0 ± 3.24^*^
HbA_1c_ (%)	3.2 ± 0.16	6.3 ± 0.26^*^	9.8 ± 0.17^*^^#^	11.0 ± 0.23^*^
Heart rate (bpm)	460.0 ± 20.17	442.0 ± 15.26^*^	414.0 ± 22.37^*^^#^	418.0 ± 18.28^*^
LV mass (g/kg)	138.6 ± 10.52	156.3 ± 9.23^*^	165.2 ± 9.42^*^^#^	165.9 ± 10.52^*^
Heart weight/tibia length (mg/mm)	0.08 ± 0.01	0.07 ± 0.03^*^	0.06 ± 0.01^*^^#^	0.6 ± 0.03^*^
EF%	68.2 ± 9.82	61.4 ± 9.43^*^	55.4 ± 8.35^*^^#^	52.1 ± 10.08^*^
FS%	38.3 ± 2.6	30.3 ± 5.7^*^	25.6 ± 4.8^*^^#^	22.4 ± 4.2^*^
E velocity (m/s)	0.94 ± 0.23	0.89 ± 0.26^*^	0.94 ± 0.33^*^^#^	0.96 ± 0.29^#^
A velocity (m/s)	0.58 ± 0.21	0.48 ± 0.15^*^	0.41 ± 0.18^*^^#^	0.42 ± 0.25^#^
E/A ratio	1.18 ± 0.04	1.01 ± 0.08^*^	0.96 ± 0.12^*^^#^	0.91 ± 0.13^*^
IVRT (ms)	17.51 ± 0.42	22.24 ± 0.25^*^	26.13 ± 0.82^*^^#^	26.15 ± 0.36^*^
LV diastolic posterior wall thickness (mm)	0.80 ± 0.22	0.91 ± 0.18^*^	1.12 ± 0.19^*^^#^	1.10 ± 0.13^*^
LV systolic posterior wall thickness (mm)	1.27 ± 0.47	1.32 ± 0.62^*^	1.43 ± 0.75^*^^#^	1.48 ± 0.61^*^
Intraventricular diastolic septum diameter (mm)	0.78 ± 0.31	0.82 ± 0.63^*^	0.99 ± 0.35^*^^#^	1.0 ± 0.50^*^
Intraventricular systolic septum diameter (mm)	1.30 ± 0.42	1.54 ± 0.53^*^	1.60 ± 0.42^*^^#^	1.58 ± 0.61^*^
LV diastolic internal diameter (mm)	3.54 ± 0.98	4.01 ± 1.01^*^	4.65 ± 1.23^*^^#^	4.57 ± 2.00^*^
LV internal systolic diameter (mm)	2.14 ± 0.86	2.88 ± 0.62^*^	3.12 ± 0.46^*^^#^	3.04 ± 0.62^*^
LV diastolic vol (uL)	62.14 ± 9.14	68.25 ± 10.32^*^	73.52 ± 8.46^*^^#^	73.21 ± 9.37^#^
LV systolic vol (uL)	60.11 ± 8.56	64.021 ± 9.21^*^	73.20 ± 10.43^*^^#^	70.13 ± 10.27^#^

BW (body weight), BG (blood glucose), Left ventricular (LV) mass, E/A ratio, percent ejection fraction (EF), percent fractional shortening (FS), LV end diastolic diameter (LVEDD), heart weight/tibia length.

* Ctrl data were similar at 4W and 8W (^*^p < 0.05 Ctrl vs. STZ or OVE26;

# *p < 0.05 STZ 4W vs. STZ 8W), n = 12, mean ± standard error of the mean (SEM)*.

### Diabetic mice displayed alterations of inflammatory cytokine mrnas in the heart

Inflammation plays an important role in diabetes-induced cardiac pathogenesis (50). Consistent with this notion, the expressions of TNF-α, IL-6, and IL-1β pro-inflammatory cytokines were substantially increased in diabetic hearts as compared with control hearts (Figures 1A–C). IL-4, a cytokine considered anti-inflammatory, was significantly downregulated in the diabetic group as compared to the non-diabetic group (Figure 1D).

**Figure 1:** mRNA expression of inflammatory molecules in diabetic mice heart tissue. **(A)** TNFα level, **(B)** IL-6 level, **(C)** IL-1β level, **(D)** IL-4 level in the left ventricular hearts. Data are expressed in mean ± SEM (^*^p < 0.05 as biological significant level, Ctrl vs. STZ), *n* = 6.

### B cell infiltration decreased in the diabetic mouse heart

Evidence showing the involvement of inflammation in diabetes has largely focused on inflammatory cytokines and reactive oxygen species (51). However, the role of the immune system and specifically immune regulation by B cells during the development of DCM is unknown. In order to confirm the effect of diabetes induction by STZ on the B cell numbers in the heart, we performed an immunohistochemical analysis. Figures 2A,C showed a significant decrease in the number of cells positive for CD19, a biomarker for normal and neoplastic B cells (52), in the diabetic hearts as compared to control. To support this finding, we used staining for CD21, another B cell marker (53). The number of CD21 positive cells was also significantly decreased in diabetic hearts at 4 and 8 W after STZ injection (Figures 2B,D). Immunoblotting confirmed that the expression levels of CD19 and CD21 were significantly decreased in diabetic hearts as compared to control (Figures 2E,F). Next, we performed flow cytometry analysis of cells infiltrating the heart tissue obtained from control and diabetic WT mice. At 4W after diabetes induction, the frequency of CD19^+^ B cells among leukocytes (CD45^+^) in heart tissue decreased from 20.4 to 8.9% and then further decreased to 4.9% at 8W after diabetes induction (Figure 2G; gating strategy is shown in Supplementary Figure 1).

**Figure 2:** Immunohistochemical analysis of B cell expression and quantification in diabetic mice heart. **(A,C)** CD19 expression and quantification, **(B,D)** CD21 expression and quantification. **(E,F)** Immunoblot representation of B cell markers CD19 and CD21 expression and quantification. **(G)** Flow cytometric analysis of B cell markers expression at 4W and 8W in control and diabetic heart mice. Data are expressed in mean ± SEM (^*^p < 0.05 as biological significant level, Ctrl vs. STZ), *n* = 6. ^#^*p* < 0.05 as biological significance level, STZ 4W vs STZ 8W.

To assess whether a decrease in the number of the B cells observed in the diabetic hearts could be due to STZ toxicity or not, we analyzed these B cell numbers in the hearts from OVE26 mice. Interestingly, immunostaining and immunoblot analysis showed a significant decrease in B cell number in heart tissues (Figures 2A–F), arguing that the observed decrease is not due to STZ toxicity, but because of diabetes condition.

To further determine whether B cells may play an important role for cardiac function, we induced diabetes on muMT^−/−^ mice (mice lacking B cells) and analyzed heart function. Interestingly, compared to WT mice, muMT^−/−^ mice show a decrease in cardiac contractile function under basal conditions and an exacerbation of contractile dysfunction after diabetes induction (Supplementary Table 1).

### Presence of B cell was not affected by diabetes induction in organs other than heart

Next, we determined whether STZ-induced diabetes affects the presence of B cells number in organs other than heart. CD19 immunostaining shows no alteration in the numbers of circulating, splenic, kidney, or bone marrow B cells in diabetic animals as compared to control (Figures 3A–H). Similar results were found in OVE26 mice. Flow cytometric analysis confirmed the lack of significant changes of B cells number in circulation and spleen (Figures 3I,J). These data clearly indicate that diabetes selectively attenuates B cell numbers in the hearts.

**Figure 3:** B cell expression was not affected by diabetes induction in other organs compared to heart. Immunohistochemical analysis of B cell CD19 expression and quantification in kidney **(A,C)**, spleen **(B,D)**, blood **(E,G)**, and bone marrow **(F,H)**. **(I,J)** Flow cytometric analysis of B cell CD19 expression and quantification in blood and spleen. Data are expressed in mean ± SEM, *n* = 6.

### Allograft inflammatory factor-1 expression decreased in diabetic hearts

In order to understand the mechanism behind the decrease in the B cells number in diabetic hearts, we first looked at the B cell inflammatory genes that might be responsible for B cells homing to the heart. In Figures 4A–C, an Affymetrix microarray showed that the most top downregulated B cell inflammatory gene is allograft inflammatory factor-1 (AIF-1). AIF-1 was 1.5- and 2-fold downregulated in STZ 4 and 8 W, respectively. Moreover, the Ingenuity Pathway Analysis (IPA) analysis of the microarray data indicated that AIF-1 is involved in cardiovascular function and inflammatory responses (Supplementary Figure 2A), further compelling us to focus on this gene. IPA analysis demonstrated the network of interactions related to AIF-1 with several inflammatory and apoptotic genes (Supplementary Figure 2B).

**Figure 4:** B cell inflammatory gene expression in diabetic mice heat. **(A)** Heat map represents data of differentially expressed genes in STZ-treated diabetic mice (4D: STZ 4W, 8D: STZ 8W) compared with Ctrl (4C: Ctrl 4W, 8C: Ctrl 8W). Genes were identified by performing *t*-tests on the large original dataset and comparing each diabetic group with the relative ctrl group. Features with significantly different expression (*p* < 0.05) were included. The heat map is organized with individual samples arranged along the Y-axis, and the relative ratios of expression are indicated by color. Color intensity is scaled as highest expression corresponding to bright red and the lowest expression corresponding to bright blue. Genes that are up- or down-regulated ≥1.5-fold are displayed in red (up-regulation) and blue (down-regulation) respectively. **(B)** 1.5-fold change B cell inflammatory gene at 8W heart vs. Ctrl heart, **(C)** AIF-1 expression from microarray data, **(D)** qPCR mRNA expression of AIF-1, **(E,F)** immunoblot expression of AIF-1 and quantification, **(G,H)** immunohistochemical analysis of AIF-1 and quantification. Data are expressed in mean ± SEM (^*^p < 0.05 as biological significant level, Ctrl vs. STZ), *n* = 6. **(I,J)** A20 B cell line incubated with low glucose (LG; 5 mM) or high glucose (HG; 35 mM) for 48 h. High glucose affects B cell marker expression. (^*^p < 0.05 as biological significant level, LG vs. HG), *n* = 4. ^#^*p* < 0.05 as biological significance level, STZ 4W vs STZ 8W.

A diabetes-induced decrease in AIF-1 gene expression in heart tissue was confirmed using quantitative PCR (qPCR) analysis. AIF-1 expression was significantly reduced at 4 W (by 40%) and further decreased at 8 W (by 69%) after diabetes induction as compared to control (Figure 4D). Next, we determined whether the changes in AIF-1 protein expression were similar to those for AIF-1 mRNA. Protein was extracted from the same hearts as used to purify RNA and subjected to the immunoblot analysis with an AIF-1-specific antibody. Figures 4E,F indicate that AIF-1 protein expression also significantly decreased in diabetic hearts following the pattern of mRNA expression.

To confirm our data, serial sections from mouse hearts at 4 and 8 W were immunohistologically examined with an anti-AIF-1 antibody. Consistent with the data on protein expression levels determined by immunoblot analysis, the results of immunohistology showed a significant decrease in AIF-1 protein at 4 W and further reduction at 8 W after diabetes induction (Figures 4G,H). Overall, our results demonstrate that AIF-1 expression decreased in parallel with the number of B cells in the diabetic hearts, thus indicating that AIF-1 may play a role in B cells homing into diabetic hearts.

### Diabetes decreased the number of AIF-1-positive B cells in the heart tissues

The effect of AIF-1 on B cell homing into the hearts has not been reported previously, nor has the functional role of B cells in the diabetic heart pathophysiology been explored. Our data showed that CD19 and AIF-1 are expressed in nondiabetic hearts tissues (Figures 5A,B), and their expressions are significantly attenuated at 4 and 8 W after diabetes induction. To analyse whether B cells migrate to AIF-1-expressing heart tissue, double immunofluorescence was performed to examine the co-localization of AIF-1 with B cell marker-CD19 in heart tissues derived from diabetic or nondiabetic mice (Figure 5C). Immunofluorescence staining showed a significant decrease in AIF-1^+^/CD19^+^ co-localization in the diabetic heart tissues as compared with the nondiabetic ones. Figure 5D shows the number of AIF-1^+^/CD19^+^ double positive cells in heart tissues from nondiabetic and diabetic mice. In samples from nondiabetic hearts, there are 34 ± 5.2 AIF-1^+^/CD19^+^ cells/mm^2^, whereas AIF-1^+^/CD19^+^ cells numbered in diabetic mice 10 ± 3.5 in diabetic mice at 4 W and 4 ± 2.8 cells/mm^2^ at 8 W. These results indicate that the number of AIF-1-positive B cells in the heart is higher in control mice, but co-significantly decreases in diabetic mice hearts.

**Figure 5:** Diabetes induction decreased AIF-1 interaction with B cells in heart mice heart. **(A,B)** Presence of CD19 (first row) and AIF-1 (second row) positive cells in control mice hearts and downregulation of CD19-positive cells as well as AIF-1-positive cells in diabetic mice hearts were observed as compared to control. alpha-actinin antibody was used to show the cardiomyocytes in the image. CD19 and AIF-1 antibodies (green), alpha-actinin antibody (red), DAPI (blue). **(C)** Immunofluorescence analysis for co-localization of CD19 and AIF-1 in mice heart. **(D)** Co-localization quantification. Data are expressed in mean ± SEM (^*^p < 0.05 as biological significant level, Ctrl vs. STZ), *n* = 6. ^#^*p* < 0.05 as biological significance level, STZ 4W vs STZ 8W.

### AIF-1 promotes B cell homing into the heart tissues

First, we assessed the effect of hyperglycemia on AIF-1 expression. Figures 6A,B show that high glucose decreased the expression of AIF-1 in H9C2 cells. To further gain more insight into the role of AIF-1 in B cell expression and migration, H9C2 cells in the presence of high glucose were transfected either with an empty vector or an AIF-1 expression plasmid. Figures 6C,D shows that the B cell migration in this system is regulated by AIF-1 expression, as B cells rapidly migrate to AIF-1 transfected H9C2 cells, but not to control cells transfected with an empty vector (Figures 6C,D). These data suggest that AIF-1 promotes B cell migration under the hyperglycaemic condition.

**Figure 6:** AIF-1 overexpression promoted B cell migration in hyperglycaemic condition. **(A)** Effect of hyperglycemia on AIF-1 expression using H9C2 cell line using immunoblot. **(B)** Analysis. **(C)** The H9C2 cells were transfected either with GFP-tagged AIF-1 plasmid or a GFP-empty vector and incubated for maximum 4 h. H9C2 cells were transfected either with a GFP tagged empty vector or GFP tagged AIF-1 plasmid. A20 cells transfected with RFP tagged empty vector and plated in the upper chamber. **(D)** Quantification of B cells migrated to AIF-1-transfected H9C2 cells. Green color represents the H9C2 cells as they were either transfected with GFP empty vector or GFP tagged AIF-1 plasmid; red color represents the A20 cell line as the A20 cells were transfected with RFP empty vector. (^*^p < 0.05 as biological significant level, Empty vector vs. AIF-1 plasmid), *n* = 4.

To determine the effect of AIF-1 overexpression in an *in vivo* model, mGFP-AdAIF-1 was injected intravenously into control and diabetic mice. Table 2 shows a significant restoration of the body weight for the mGFP-AdAIF-1 injected mice, as compared to the WT STZ 8W mice that were not injected with this viral vector. Notably, the blood glucose level was to not affected by the AIF-I vector. Echocardiography data showed a significant restoration of left ventricular (LV) mass, ejection fraction (EF), fractional shortening (FS), E/A ratio, IVRT, heart weight/tibia length and other echo parameters as compared to the WT-STZ 8W mice heart. Interestingly, AIF-1 overexpression inhibited inflammation (Figures 7A–D) and increased the expression levels of CD19 and CD21 B cell markers in diabetic heart tissues as compared to the untreated diabetic mice heart tissues (Figures 8A–F). Further, flow cytometry analysis confirmed that AIF-1 overexpression increased the number of B cells in diabetic hearts as compared to the hearts of untreated diabetic mice (Figure 8G). Taken together, these data strongly suggest that AIF-1 promotes B cell homing into the heart tissues.

**Table 2:** Physiological parameters and echocardiography assessment of heart function after overexpression of AIF-1 in diabetic mice.

**Parameters**	**WT**			
	**Ctrl 8W**	**STZ 8W**	**AdAIf-1Ctrl 8W**	**AdAIf-1STZ 8W**
BG (mg/dl) or BG (mM)	120 ± 10.25 or 6.66 ± 1.27	480 ± 11.36^*^ or 26.64 ± 1.64	126 ± 11.27 or 6.99 ± 1.48	390 ± 12.45^*^^#^ or 21.65 ± 1.96
BW (g)	24 ± 2.16	19 ± 1.98^*^	23 ± 2.26	22 ± 2.20^*^^#^
HbA_1c_ (%)	3.4 ± 0.16	8.9 ± 0.24^*^	3.8 ± 0.18	4.0 ± 0.22^*^^#^
Heart rate (bpm)	454 ± 22.32	410 ± 18.32^*^	448 ± 16.48	450 ± 17.59^*^^#^
LV mass (g/kg)	133.38 ± 8.22	164.22 ± 10.19^*^	134.22 ± 9.25	133.41 ± 8.13^*^^#^
Heart weight/tibia length (mg/mm)	0.08 ± 0.02	0.06 ± 0.01^*^	0.08 ± 0.01	0.08 ± 0.02^*^^#^
EF%	62.01 ± 10.14	43.26 ± 8.48^*^	59.47 ± 9.42	60.05 ± 9.18^*^^#^
FS%	32.16 ± 7.59	20.32 ± 1.28^*^	30.08 ± 5.13	29.46 ± 4.89^*^^#^
E velocity (m/s)	0.95 ± 0.21	0.89 ± 0.26^*^	0.94 ± 0.33	0.96 ± 0.29^*^^#^
A velocity (m/s)	0.58 ± 0.20	0.42 ± 0.18^*^	0.52 ± 0.24	0.56 ± 0.21^*^^#^
E/A ratio	1.55 ± 0.21	1.00 ± 0.18^*^	1.50 ± 0.16	1.54 ± 0.14^*^^#^
IVRT (ms)	17.51 ± 0.42	25.35 ± 0.48^*^	18.26 ± 0.32	16.05 ± 0.26^*^^#^
LV diastolic posterior wall thickness (mm)	0.82 ± 0.16	1.14 ± 0.27^*^	0.84 ± 0.14	0.83 ± 0.21^*^^#^
LV systolic posterior wall thickness (mm)	1.26 ± 0.45	1.42 ± 0.35^*^	1.22 ± 0.41	1.24 ± 0.38^*^^#^
Intraventricular diastolic septum diameter (mm)	0.75 ± 0.22	0.98 ± 0.47^*^	0.72 ± 0.37	0.74 ± 046^*^^#^
Intraventricular systolic septum diameter (mm)	1.32 ± 0.38	1.62 ± 0.43^*^	1.33 ± 0.42	1.58 ± 0.61^*^^#^
LV diastolic internal diameter (mm)	3.52 ± 0.84	4.59 ± 1.23^*^	3.65 ± 1.20	3.55 ± 1.56^*^^#^
LV internal systolic diameter (mm)	2.17 ± 0.38	3.15 ± 0.27^*^	2.21 ± 0.52	2.20 ± 0.48^*^^#^
LV diastolic vol (uL)	61.21 ± 8.22	72.78 ± 9.60^*^	62.34 ± 8.24	62.49 ± 10.36^*^^#^
LV systolic vol (uL)	61.56 ± 9.17	74.01 ± 10.12^*^	60.23 ± 8.22	62.31 ± 9.31^*^^#^

BW (body weight), BG (blood glucose), Left ventricular (LV) mass, E/A ratio, percent ejection fraction (EF), percent fractional shortening (FS), LV end diastolic diameter (LVEDD), heart weight/tibia length (

* p < 0.05 Ctrl vs. STZ; ^*^p < 0.05 AdAIF-1Ctrl vs. AdAIF-1STZ;

# *p < 0.05 STZ vs. AdAIF-1STZ), n = 12, mean, standard error of the mean (SEM)*.

**Figure 7:** AIF-1 overexpression decreased inflammation in diabetic mice hearts. **(A)** TNFα level, **(B)** IL-6 level, **(C)** IL-1β level, **(D)** IL-4 level. Data are expressed in mean ± SEM (^*^p < 0.05 Ctrl vs. STZ; ^#^*p* < 0.05 STZ vs. AdAIF-1 STZ), *n* = 6.

**Figure 8:** AIF-1 overexpression promoted B cell homing in diabetic mice hearts. **(A,C)** Immunohistochemical of CD19 expression and quantification, **(B,D)** immunohistochemical CD21 expression and quantification, **(E,F)** immunoblot analysis of B cell markers (CD19 and CD21) and quantification. **(G)**. Flow cytometric analysis of B cell number in diabetic hearts after AIF-1 overexpression as compared to diabetic hearts. Data are expressed in mean ± SEM (^*^p < 0.05 Ctrl vs. STZ; ^#^*p* < 0.05 STZ vs. AdAIF-1 STZ), *n* = 6.

## Discussion

Chronic hyperglycaemia results in the release of enzymes that cause inflammation leading to cardiac dysfunction and myocardial cell death (54) and eventually to DCM. Several factors have been shown to contribute to the development of DCM and cardiac failure. Humoral immunity plays important role in heart disease and cardiac failure (55). Therefore, understanding the mechanisms underlying type 1 diabetes-associated pathophysiology and its effect in cardiac disease are pertinent for the development of therapeutic interventions to curb this epidemic. The results of this study demonstrate for the first time that the expression level of B cell markers and the B cell number are decreased in the diabetic heart tissues and this downregulation is associated with the downregulation of AIF-1 expression. Interestingly, overexpression of AIF-1 promoted B cell homing into the heart tissues, which in turn prevented cardiac dysfunction-mediated by type 1 diabetes induction. As a result, cardiac inflammation was significantly reduced in AIF-1 overexpressed diabetic hearts due to the increase of B cell immune responses, which result in a preserved cardiac function. In the present study, AIF-1 overexpression after the insult of diabetes reduced the extent and progression of cardiac dysfunction and enhanced cardiomyocyte survival.

Consistent with previous studies (56–58), injection of STZ led to the significantly increased blood glucose levels and decreased body weight. Hyperglycaemia induced an increase in the inflammatory response, which in turn leads to diabetic complications. The evidence for involvement of inflammation in diabetes has largely focused on inflammatory cytokines and reactive oxygen species (51, 59–61). However, the role of the immune system and specifically immune regulation by B cells during the development of DCM is largely unknown. Immunohistochemical staining, immunoblot, and flow cytometry assays demonstrated that the expression levels of CD19 and CD21 were significantly decreased in diabetic heart tissues as compared to control. But in our data, we have also proved that during DCM, the B cell production and development is not altered, as we found that B cell numbers are not decreased in other organs like kidney, spleen, bone marrow and blood. Previous studies showed that in type 2 diabetic patients, B cells infiltrate more in kidney (62, 63). Another study proved that marginal-zone B cells number increased in diabetes (64). Studies have also shown that in diabetes B cells number is increased in spleen and kills the beta cells in the spleen (65). But no previous data reported about the number of B cells presence in these organs during the development of DCM.

Furthermore, to understand the mechanisms behind the decrease of B cell number in diabetic hearts, we first looked at the B cell inflammatory genes that might be responsible for B cell homing into hearts. Interestingly, the microarray analysis indicated that AIF-1 was among the top differentially expressed B cell inflammatory genes that are significantly downregulated in DCM. AIF-1 is constitutively expressed in monocytes/macrophages and T cells, but no published study has shown the role of AIF-1 in B cell homing into the hearts. The network of interactions built using IPA centered on AIF-1 demonstrates the link between AIF-1 and several genes and gene products that are highly relevant to inflammation and apoptosis. AIF-1 also directly or indirectly interacts with genes and gene products that are primarily associated with the regulation of T cells and immature thymocytes production (NF-ATC3), inflammatory responses (CXCL12, IL-17A), collagen synthesis (COL1A1) and DNA replication (PCNA). The signaling pathways linked to AIF-1 are also connected to several microRNAs (mir-27, 21, 4,522, 6,835, and 6,732) that have primary biological process functions associated with the cell-cycle regulation. IPA analysis further showed that AIF-1 is connected with several network of interactions related inflammatory and apoptotic genes Bcl-2 and Bad, important apoptosis regulators (66). Our immunohistochemical and immunoblot analysis confirmed downregulation of AIF-1 expression in heart tissues following the experimental diabetes induction. It has been shown that AIF-1 is involved in the inflammatory responses and is expressed in monocytes, macrophages and T cells in the heart tissues (67). However, its role in B cell homing has not been described yet. The present study showed that AIF-1 is necessary for B cell homing in the heart tissues as assessed by immunostaining, which showed that AIF-1 is co-localized with CD19-positive cells in nondiabetic hearts and this co-localization is significantly decreased in the diabetic heart tissues. The *in vitro* migration assay confirmed that B cells migrated to hyperglycaemic H9C2 cells in the presence of AIF-1, but not in its absence. These findings are in line with the idea that AIF-1 is a key regulator for the B cell homing to the diabetic heart tissues.

Several potential mechanisms could also contribute to the homing of B cells into the heart tissues. To date, we have determined that AIF-1 is a key regulator for B cell migration using an *in vitro* culture system. Although further research should clarify the role of AIF-1 in B cell responses *in vivo*, it is quite possible that the *in vitro* culture system reflects key features of the *in vivo* situation and thus is useful for facilitating our understanding of the role of AIF-1 in B cell biology. Furthermore, mGFP-AdAIF-1 injection in a diabetic mouse model showed a significant attenuation of inflammatory markers. At the same time, injection of mGFP-AdAIF-1 increased the B cell homing into the heart tissues. Interesting, mGFP-AdAIF-1 injection showed an alleviation of cardiac dysfunction as assessed by echocardiography. This data confirmed that AIF-1 plays a key role in suppressing inflammatory responses in the diabetic heart by maintaining a normal physiological level of B-cell functions in the heart. An increase in the levels of CD19 and CD21 in the presence of AIF-I further argued that presence of AIF-1 can promote the B cell homing into the heart. Different research articles already established that inflammation is one of important pathophysiological cause of onset of DCM (68, 69). In our study we found that B cell homing leads to a decrease in inflammatory responses, which leads to an increase in anti-inflammatory marker IL-4. Our present study also stated the same result as other studies shown involvement of inflammation in the progression of cardiac dysfunctions. So, in this study we focused to attenuate the inflammation and inflammatory responses by increasing the B cell homing in DCM heart. These B cells homing further leads to downregulation of inflammation as a pathophysiological trigger. We believe that the inhibition of cardiac inflammation is due to B cell homing but not AIF-1 expression. However, the mechanisms behind this finding is not clear yet. But according to our present study and previous literature the probable mechanism can be something related to AIF-1 and chemokine interactions.

It has been shown that AIF-1 up-regulates several CC chemokine genes that could induce PBMC migration toward inflamed tissue (70) and a specific protective role of B cells has been shown to play a role in modulating the immune response under pathogenic conditions. These specific B-cell subsets can down modulate the immune response through production of anti-inflammatory cytokines (71). In our model, we hypothesize that AIF-1 releases chemokines that will promote B cell homing and activation in diabetic heart tissue which in turn will release anti-inflammatory cytokines. Although further work is needed to clarify the molecular mechanism of AIF-1 action in our diabetic model. It is well known that NF-κB is clearly one of the most important regulators of pro-inflammatory gene expression. However, it has also been suggested that NF-κB activation in leukocytes during the resolution phase of the inflammatory process results in upregulation of anti-inflammatory genes and induces leukocyte apoptosis (72). NF-κB activation is also involved in regulation of cell survival and modulates matrix metabolism by regulating Matrix Metalloproteinase (MMP) synthesis (73). Thus, activation of the NF-κB signaling cascade in the injured heart involves various cell types and affects multiple parallel processes with an essential role in cardiac injury and repair.

Our next step is the identification of AIF-1 targets that are critical for the modulation of the cardiac B cell immune responses. But also we considered that as we used the mGFP-AdAIF-1 injection in early onset of diabetes, that could be a limitation of this study to rescue the diabetic cardiomyopathy phenotype. Our future approach is to inject cardiac-specific mGFP-AdAIF-1 in mice model which will be more beneficial with respect to clinical and translational relevance.

## Conclusion

In conclusion, the reduced B cell homing into the heart tissues might be the one of the most important factors causing DCM. To the best of our knowledge, we are the first to report a correlation between the AIF-1 expression and B cell infiltration; both of which are downregulated during the development of DCM.

The biological function and the mechanism of action of AIF-1 have not been fully elucidated. Future studies are in progress to study the level of B cell distribution during DCM and the effects of AIF-1 in the restoration of systemic B cell number. An AIF-1 transgenic model may attenuate the cardiac remodeling by restoring B cells during the development of DCM. Furthermore, AIF-1 also exhibits a certain therapeutic potential *in vivo* and *in vitro* (74). A previous study has confirmed the clinical importance of AIF-1 upregulation in several conditions such as systemic sclerosis, rheumatoid arthritis, and transplant-related arteriosclerosis (75, 76). To sum up, further research on the role of AIF-1 in B cell homing included, during the development of DCM is warranted.

## Author contributions

AS designed and performed experiments, analyzed data, and wrote the manuscript. SS and AA contributed to performing the experiments and correcting the manuscript. AK isolated cells from the heart tissues and performed flow cytometry. SA contributed to performing the experiment and analysis for microarray. AT discussed the results and participated in editing the manuscript. KR is a guarantor of the manuscript, designed the experiments, supervised all experiments, checked and edited the manuscript.

### Conflict of interest statement

The authors declare that the research was conducted in the absence of any commercial or financial relationships that could be construed as a potential conflict of interest.

## Supplementary material

Supplementary Figure 1 Gating strategy. Heart tissues from control and diabetic mice were stained with CD4, CD8, CD45, and CD19 antibodies and analyzed with flow cytometry, *n* = 6.

Supplementary Figure 2 IPA analysis. **(A)** Functional analysis of AIF-1 from microarray of mice heart tissue. **(B)** AIF-1 gene network by IPA analysis.

Supplementary Table 1 Physiological parameters and echocardiography assessment of heart function in B cell knock out muMT mice. BW (body weight), BG (blood glucose), Left ventricular (LV) mass, E/A ratio, percent ejection fraction (EF), percent fractional shortening (FS), LV end diastolic diameter (LVEDD), heart weight/tibia length (^*^*p* < 0.05 muMT Ctrl vs. muMT STZ), *n* = 12, mean ± standard error of the mean (SEM).
